RETRACTED

# Analysis of the Effectiveness of International Law in Global Environmental Relations from the Perspective of International Institutional Theory

**DOI:** 10.1155/2022/1505040

**Published:** 2022-08-28

**Authors:** Zeyang Yu

**Affiliations:** Department of International Relations, College of Asia and the Pacific, Australian National University, Canberra 2600, ACT, Australia

## Abstract

Since the 1970s, mankind has become increasingly sensitive to major world environmental protection issues, and the globalenvironmental protection laws and regulations system formed to deal with suchspecific issues has rapidly expanded in scope and depth. From the initial environmental issues in the study of international relations theory to the development of environmental issues in the study of global governance, and then the concept of global environmental governance came out and developed rapidly. This trend provides a desire to deal with many environmental protection issues and various issues related to worldenvironmental protection issues. But are these wishes real? We must also doubtthe rationality of the legal systems of various countries that have been formedand fought to deal with all environmental protection relations, especially theworld environmental protection issues. Today, the world environmental problemhas formed a relatively perfect academic field. The concept theory of globalproblems starting from ecological problems has moved from ecological problemsto world governance problems. With the introduction and rapid improvement ofthe concept of world ecological problems. The articlestarts from the role of non-state actors in the original internationalframework, further expands and deepens, and presents a multiangle andall-round perspective, showing that international law can still play a crucial role in the settlement of international environmental problems. It not only caters to the needs of the current international situation and development but also provides forward-looking guidance for future environmental governance at the global level.

## 1. Introduction

The research scope of global impact of environmental issues is also relatively late, which is much lower than the research field ofwar and conflict. It gradually attracted people's attention, which reflected the increasingly serious environmental protection problem at that time. The Canadian historian Arnold Joseph Toynbee once said: if people want toprevent its damage, they can consider the harm it brings from now on, and cannot let it happen again. I believe this can be achieved through globalcooperation.The study of environmental issues in international relations, and the study of global environmental governance, is a response to this concern [1]. With industrialization, global resource consumption has risen dramatically, as shown in Figure 1, and the consumption of these resources is itself a problem of environmental impact, not to mention the environmental impact of the massive pollution that results from its consumption, so environmental issues have caught the research eye of international relations [2]. With the gradual deepening of globalenvironmental governance research, global environmental governance theory hasbecome a system analysis paradigm advocated by researchers in the fields ofglobal relations and environmental policy. It is the common pursuit of allmankind to build a reasonable and feasible global environmental governancesystem.

RETRACTED

The validity of international law is an importanttheoretical issue in international law and one of the general norms ofinternational law. In international justice, the ability to invoke and applylaws is also the main symbol of the effectiveness of international law. According to the summary of the researchers,the main theories based on the utility of international law include the theoryof natural law, the theory of basic rights, the theory of common will, thetheory of state self-restraint, the theory of sacredness of international contracts,the theory of international relations, and the theory of state needs [3]. However, no matter which theory is adopted, itspurpose proves that international law is reasonable from a certain side orangle. Today, when people discuss the concept of validity in international law,they should first examine the validity period of treaties, whether parties canperform treaties and whether violations of treaties can be effectivelypunished. Compliance with international law is always measured by general legalnorms [4]. However, in the case of general principles of law, if they cannot be invoked by international judicial bodies and become declaratory or otherwise, their validity is greatly reduced or questioned [5]. It is generally believed that in international disputes, general principles of law have little chance of being directly invoked. Despite this, Zheng Bin believes that from a judicial point of view, it cannot be denied that general principles of law have a higher value than custom and treaties; for these principles provide the judicial basis for treaties and custom and control their interpretation and application [6]. This development offers hope for the resolution of numerous environmental problems, including the range of challenges associated with global environmental change. However, is this hope realistic? This calls for questioning the effectiveness of the international legal regimes that have been established or are being worked on to address various environmental issues, particularly global environmental issues [7].

RETRACTED

The study of the effectiveness of international lawmust face the following two difficulties. First, due to the key role of powerand interests in determining global behavior, has the compliance with globallaws and regulations seen by people completely excluded the results of the two?Second, if an international treaty or system can change behavior, what factorsshould those actors and system designers who participate in the negotiation payattention to to to improve the maximum efficiency of the system? Therefore,after analyzing the actual cases of global environmental relations, this paperpoints out that the international law system can still play a key role indealing with global environmental issues, and there are some important reasonsthat can enhance or weaken this effectiveness. It is of great significance for global environmental issues to be addressed in a truly international perspective.

## 2. Theory

### 2.1. Validity of International Law

There can be many ways to study the validity of international law, but it does draw nourishment from the legal theory of the international system. It is a more appropriate and reasonable way. When it comes to general principles of law in international law, it is always customary to refer to the “general principles of law” applied by the International Court of Justice within the meaning of Article 38, paragraph 1 (c), of the Statute of the Court, i. e., those “general principles of law” recognized by civilized nations. The meaning of this phrase was once the subject of lively discussion. Nowadays, scholars' understanding of general principles of law in international law has evolved considerably [8]. Many people have adopted a more pragmatic approach andno longer limited their understanding of the general principles of law to the “general principles of law” within the meaning of Article 38 (1) (c)of the statute of the International Court of justice. However, in addition torecognizing the “general principles of law” derived from the domesticlaws of civilized countries and the “general principles of law” derived from the domestic laws of civilized countries. They have beenincorporated into the general norms of international law. The basic structure of international law is shown in Figure 2.

### 2.2. Definition of the Effectiveness of International Law

The current jurisprudence is mainly a substitute for the modern Western philosophy of law, and its object of study is “general law”, that is, the whole legal field including international law and all the laws of the past and the present. product of a particular historical era, i.e., it matured before the emergence of international law. This means that jurisprudence based on the background of regimes and ruling groups has limitations in studying and grasping the rules of international society under anarchy [9]. It is difficult to find the theoretical support forthe validity of international law from the general precedents guiding domesticlaw. Although international law has been classified into the category of “general law,” the theory of “legal effect” injurisprudence has not been directly applied to international law through itseffect on international law. Therefore, the definition of the validity of international law is faced with the problem of lacking the support of “international jurisprudence,” but it is not willing to simply look for inappropriate answers from general jurisprudence [10]. International Convention refers to a kind ofpolitical, economic, trade, science, and technology, etc. in variouscountries through international conventions or multilateral treaties.Agreements are generally open and non Contracting States may participate inthem at any time before and after their entry into force. Some conventions areproposed by professional international conferences, such as those listed in Table 1.

RETRACTED

### 2.3. Validity of General Legal Principles in International Tribunals

It is only natural that the permanent and international courts do not have many opportunities to apply general principles of law, because, as a rule, international treaties and customary law are sufficient to provide the necessary basis for decisions. Moreover, since scholars are deeply divided on general principles of law, most notably because of their ambiguity, judges enjoy a great deal of discretion, and sovereign states are reluctant to leave their fate to the “whim” of a few judges who cannot foresee the outcome of a case [11].

One principle that has been invoked by the ICJ and is extremely important is the principle of good faith. “A very few international jurisprudence has based its decisions on the principle of equity, and the Permanent Court of International Justice has based its decisions on the principle of equity in cases concerning damages.” The use of equitable principles as a basis for the ICJ's decisions began in the North Sea Continental Shelf Case [12]. The principle of justice has been adopted and hasbecome the main basis for the judgment of the International Court of justice.The International Court of justice held in its trial of the North Seacontinental shelf case in 1969 that “as a legal concept, fairness is adirect reflection of the concept of justice.” It is a “general principle of law that can be applied directly, like law.” The classification of legal principles is shown in Table 2.

RETRACTED

### 2.4. Effectiveness of International Law in Environmental Relations

When it comes to the effectiveness of international law, itis not uncommon to encounter difficulties: for example, legal actors can opposethe consequences of institutional arrangements at the beginning; even, theregulations are sometimes broken because of the difference in legal priority;or the international political system and knowledge base formed by themechanism will be doubted. Of course, the more such problems arise, the moredifficult it will be to realize the effectiveness of international law.However, the occurrence of a difficult situation does not mean thatinternational law is useless to the actions of individual individuals or groupsin the global community, nor does it mean that it is powerless or evenirrelevant in dealing with environmental issues at the global level. If it is said that the international legal system can notonly maintain its original face in complex environmental relations, but alsoexert a great impact on the activities of individuals or groups, it can beinferred that under a more favorable environment, it may produce effects orbecome more powerful. To this extent, the validity problem is only a degreeproposition, not an incomplete proposition.

After the 20th century, with the advancement of science and technology, economic development, and the growing seriousness of environmental problems, the international relations community also began to pay attention to environmental issues, such as the emergence of a large number of new journals focusing on environmental issues, and the emergence of the GreenTheory branch of international relations theory on environment and ecology, which studies environmental issues in international relations through different research perspectives [13].

The increasing trend of world economic integration has deepened the international division of labor, and the economic ties between countries have become closer, so international direct investment has become the main form of a country's participation in international economic competition [14]. This also makes mankind rethink the economicdevelopment model that has a devastating negative impact on the environment, while paying more attention to the analysis of the elements and pathwaysthat affect the ecological environment. When environmental relations also have an international perspective and begin to face cross-border environmental impacts, the issue of the relationship between the international perspective and environmental relations enters the research horizon. An in-depth study of the issue of environmental relations from an international perspective first reveals the main sources of global environmental problems as shown in Figure 3 below [15].

RETRACTED

## 3. Environmental Issues in International Relations' Research

After the 20th century, due to the improvement ofscience and technology, the development of national economy and theincreasingly serious environmental protection problems, the internationalrelations community also began to pay attention to international environmentalprotection problems, such as the emergence of a large number of new journals oninternational environmental protection issues and the emergence of green theorybranches on environmental protection issues and ecological construction inrelevant international theories, and the emergence of the GreenTheory branch of international relations theory on environment and ecology, which studies environmental issues in international relations through different research perspectives [16], as shown in Figure 4.

### 3.1. Neo-Liberal Institutionalist International Relations' Scholars Propose a Theory of International Mechanisms

First, neoliberal institutionalist scholars of international relations developed theories of international mechanisms to analyze environmental problems. In 1977, Joseph S. Nye and Robert o. Keohane publishedhis book power and inter dependence, which discussed environmental issues andbelieved that “for the federal, international systems and ecosystemsaffected by the continuous growth of enterprise waste, it is necessary to adoptcommon measures to prevent disasters.” In 1983, Ernst Hass furtheremphasized the natural evolution theory and the theoretical direction ofenvironmental development of international institutional theory, pointing outthat ecology is not only a natural theory, but also the most important theory reflectingthe development trend of global market economy and society. Therefore,international relations theory has become the basic theoretical perspective ofworld environmental governance [17].

### 3.2. The Green Turn in International Political Economy

Considering economic input may also reduce theeffectiveness of the international legal system. In 1978, DANNIS pirages wrote in global economicpolitics: new contents of international relations that international politicaleconomy should evolve into global political economy, and its scope shouldinclude the interaction between policies and economic activities of the wholeworld region, covering a wide range of issues. In 1989, the British economistDavid pierce clearly put forward the concept of “green economy” forthe first time in his research report “green economy blueprint.” In 2008, at the time of global financial crisis and macroeconomicdepression, the United Nations Environment Programme (UNEP) launchedinitiatives such as “green economy” and “Green New Deal” around the world, and produced a large number of important researchresults on environmental protection and ecological construction. Ininternational political economy [18].

RETRACTED

### 3.3. Safety Research Begins to Focus on Environmental Issues

In 1987, the 42nd session of the United Nations General Assembly unanimously adopted the famous report of the Brundtland Commission, our common future, which emphasized that the definition of security must be expanded beyond political and military threats to national sovereignty to include environmental degradation and the destruction of development conditions. The report also pointed out that the concept ofoverall security should be extended to political and military threats tonational sovereignty and include damage to environmental degradation andeconomic conditions. The report adopted the concept of “environmentalsecurity” for the first time. The report clearly points out: “thewhole security theory traditionally defined - from the political and militarythreats to national sovereignty - should be extended to military threatsincluding greater environmental pressure... Regional, national, regional andglobal.” The end of the cold war and the change of the world environmentalprotection situation have promoted the international academic circles to payattention to the environmental security issues. The scholar Rita Floyd pointedout in her recently published Environmental Security Research Book EnvironmentSecurity: approaches and issues that environmental security methods are oftenscattered, lacking integrity and integration, and integrating ecologicalsecurity issues, involving water resources, food, sustainable development,environmental resources, and climate change [19].

From the general trend of the development of international perspective, the environmental issues of developed countries have been the most important market for global environmental relations, however, the future growth of trade cooperation between developed countries and China has been relatively limited, which is due to the lack of economic growth in developed countries after the financial crisis, the United States is slightly better than other developed countries environmental issues in about 2% to 3%, while the United Kingdom, Germany, France, Japan, and other developed countries generally deal with trends lower than the United States, as shown in Figure 5.

### 3.4. Summary of Key Factors Affecting the Effectiveness of International Law

The effectiveness of international law does notentirely stem from its external “coercive force,” but also from manyother aspects. These various factors directly affect the effectiveness ofinternational law, thus making other aspects of the legal system that play a leadingrole between rights and laws relatively single. The influence of international law capacity canbe generally divided into two categories: endogenous factors and exogenousfactors. It is now necessary to study the use of these key factors tostrengthen or reduce the role of legal relations between the two parties indetermining the influence of national actors in the world [20].

RETRACTED

#### 3.4.1. Structure of the Problem to Be Solved

Because the structure of the problem itself isdifferent, the legal system will always deal with some problems more simply andefficiently than other problem systems. “Collaboration” issues areeasier to handle than “collaboration” issues. Therefore, it is muchmore effective to control the transboundary movement of hazardous wastes thanto control the transboundary air. Therefore, in terms of controlling thecross-border air, all Member States believe that although other Member Statesrelease pollution without restriction, the pollution emissions unilaterallycontrolled by themselves do not fundamentally promote the overall environmentalprotection management, Even their own unilateral expansion of pollutionemissions has not had a decisive impact on the overall environmental qualitymanagement. Once they believe that the unrestricted discharge of pollution inother countries will be detrimental to the overall environmental protectionmanagement, or if their unilaterally expanded pollution discharge does not havea decisive impact on the overall environmental quality, the effectiveness ofthe legislative mechanism will be seriously damaged. Moreover, problemsinvolving many actors are also more difficult to solve than those involvingindividual actors. For example, it is much more difficult to formulate laws andregulations to maintain the international climate system than to protect theearth's ozone layer from damage. Moreover, when actors are willing to join amechanism or continue to interact indefinitely, their joint motivation isstronger than when there is a short-term relationship. For example, the globallegal mechanism for Antarctic governance has more opportunities to promoteeffective long-term cooperation, rather than through participation inshort-term agreements for the development of limited resources.

#### 3.4.2. Attributes of the International Legal System

The characteristics of the international legal system willgreatly affect its effect. Therefore, the difficulty of amending laws andregulations plays a decisive role in its rationality. The polar bear protectionagreement signed by several small northern countries in 1973 made clear thefeasibility of the reform of laws and regulations, but only proposed that “signatory countries may wish to negotiate changes to the agreement”. In contrast, the 1959 Antarctic Treaty, which forms the core of the AntarcticTreaty System, clearly stipulates a procedure for amendment, requiring allparties to the negotiations to “agree unanimously” before makingamendments. The various requirements of this revision process obviouslyrestrict members in different ways. Moreover, although most countries approveof the amendment process, the adoption of different sanctions against countriesthat attempt to violate the law will have an important impact on theeffectiveness of the provisions of the Convention. The Antarctic conventionsystem requires “consistency rules”; regulations governing trade inendangered species require “a two-thirds majority of the participantsparticipating and voting.” However, the last change is much lessmandatory, giving Member States more opportunities to violate this rule andreducing its effectiveness. In short, the regime always needs to establishreasonable legal provisions to deal with violations, and usually at the cost ofpunishment. In the judicial systems of various countries in the world, thesepunishments are usually manifested as the result of the tension of thepolitical interests or international prestige caused by the violation of thesystem, which also greatly frustrates the will and actions of political actorsagainst the violation of the system.

RETRACTED

#### 3.4.3. The Broader Context behind the System

Improving our understanding of the effectiveness of international law requires addressing the plurality of issues that come before us. The constitutional system cannot operate in a vacuum; thebroader political environment, such as economics and Biophysics, also has moreimportant factors for their ability to deal with specific environmental issues.The international law stipulates that the environment is also extremelysensitive to the broader historical background of its operation: during theperiod of macroeconomic depression or economic crisis, it may cause seriousdifficulties in dealing with global environmental protection issues; Variouspolitical and economic pressures or contradictions during the period ofimportant actors often mask the ability to deal with environmental issues, suchas the global River environmental protection mechanism effectively designed inthe Middle East and the Indian Ocean subcontinent, taking into account itspolitical relations.

## 4. Global Environmental Strategies and Actions

World environmental governance has grown into a uniqueand relatively perfect field in the field of global issues. Since the globalexploration of environmental governance has been carried out, the worldenvironmental governance has always followed the evolution of the globalobjective environmental problems and the requirements of global development. At the United Nations General Assembly Session on the global environment in July 1997, Wolfensohn, President of the World Bank, described the global environmental development strategy in general terms as follows.

RETRACTED

To propose the objectives and subjects of global environmental conferences with foresight; to link global environmental issues to the development of all sectors of the economy and to integrate them into national development strategies and policies; to propose comprehensive and rational environmental protection measures in the face of the threat of degradation or even depletion of natural resources in most countries; to develop new global energy markets and to invest in new energy products; to strengthen the professional training of staff and participants of the World Bank The World Bank's Economic Development Institute and Learning Center staff and participants in the professional training; the collaboration with the private sector in various countries to improve the practical effects of sustainable development; and the adoption of a variety of approaches to increase environmental investment at the local, regional, national, and global scales and to improve social and environmental evaluation standards. The current global environmental issues are shown in Figure 6.

The global environmental actions taken by the World Bank under the above guidelines are basically.

### 4.1. Climate Change

To enhance the competitiveness of renewable non-GHG diffusion technologies, the World Bank is working with the Global Environment Facility (GEF) and other social groups on a wide range of strategic and economic collaborations; and is preparing to establish a coal research fund so that members of the Climate Change Association are aware of their responsibilities and roles in trying to reduce the loss of entire ecosystems due to GHG diffusion. Provide World Bank-assisted countries with fair opportunities to share consumption resources and effectively use environmental protection technologies.

### 4.2. Biodiversity and Sustainable Forestry

The World Bank engages in programmatic collaboration and strategic consultation with a variety of private groups and social organizations to create productive markets for forestry with social, economic, and ecological benefits to conserve biodiversity. For example, the World Bank and the World Wildlife Fund work together to co-manage tens of millions of hectares of tropical, temperate, and boreal forestland worldwide and provide strategies for biodiversity conservation and sustainable forestry development.

RETRACTED

### 4.3. Desertification and Land Degradation

The World Bank is strongly supporting a series of recommendations and strategies adopted by the Desertification Convention that emphasize the link between poverty and land degradation, taking the most effective measures in land planning and degradation management; coordinating land use issues through integrated national policies, effectively regulating economic development in relation to international environmental action plans; and developing and implementing regulations for desert areas, using systems analysis methodology and development planning and regulation. We also develop and implement regulations for the management of desert areas, and coordinate the financial efforts of each country with the development of the world economy using the methodology of system analysis and development planning.

### 4.4. Water Resources

The World Bank has been entrusted by the United Nations to support the work of The Global Water Partnership in assisting the Commission on the Protection of Watery Places and in developing a regional ocean use plan program. The World Bank expects to comply with the Dublin Principles and invest $35 billion in water issues over the next decade.

### 4.5. Ozone Layer Destruction

The World Bank, in collaboration with the Russian government and community groups, has developed a strategy to eliminate the black market for trade in CFC-containing polymers in violation of the Montreal Protocol, and plans to phase out CFC production in Russia by the year 2000.

In addition, the World Bank, in order to effectively help countries reduce poverty and face the threat of a deteriorating global environment, has made a timely and clear case for making sustainable development a central element of its aid strategy and has decided to focus its aid core on disciplined lending and sub-lending services. The world bank is one of the institutions mainlyresponsible for the world environmental protection organization agreement(Global Environment Facility) of the Montreal draft, and is also the largestfinancing institution for the implementation of the global environment plan. Ithas formulated the project plan of the global environment department (afr-eapAfrica region ECA East Asia and Indian Ocean region lac Eastern Europe andcentral region lac MNA Middle East region and North Africa SA Southeast Asiaregion) investment programs are prepared to invest a total of $11.6 billion in 166 planned programs, mainly for environmental pollution treatment, environmental resource utilization, and funding of activities of environmental groups. Among them, the investment of funds in IEG in 2019 for the implementation of global environmental programs is shown in Table 3. The global environment facility (GEF) is anenvironmental research programme established by the world bank in 1990 to support environmentally friendly projects. The Global Environment Facility (GEF) carries out environmental projects in 183 countries and regions. Currently, the GEF mainly supports biodiversity, climate change, chemicals, and waste disposal. At present, the national environmental investmentfocuses on supporting biodiversity, climate change, chemicals and wastetreatment. At present, the United States has a total of 12.5 billion yuan ingrants and 58 billion yuan in CO financing 3690 major construction projects in165 developing countries.

RETRACTED

## 5. Conclusion

World environmental governance has developed into aunique and relatively perfect field in the field of global relations. Since therelevant theoretical research on international environmental issues has beencarried out, the issue of world environmental governance has always closelyfollowed the development trend of objective environmental problems in variouscountries and the requirements of global practice. In the paper, the effectiveness ofinternational law in the world environmental governance is investigated fromthe aspects of “whether” and “what” and less from the topic of “how” to bring into play effectiveness, which is precisely what needs to be discussed in the next section. The latter is also the issue that must be further paidattention to in the next stage of research. For example, whether the sourcerange of effectiveness is wider; What are the necessary or sufficientconditions for effectiveness; How the effectiveness of international lawaffects the actions of non-governmental actors; In the international contextwhere national power and interests drive each other, how can the governmentbetter implement the effectiveness of international law?To help China understand and deal with domestic, regional, and global environmental issues from a global perspective, and serve China's long-term strategy of participating in global governance in an all-around way.

## Figures and Tables

**Figure 1:** Global resource consumption.

**Figure 2:** The basic structure of international law.

**Figure 3:** Main sources of global environmental problems.

**Figure 4:** Impact of international trade on carbon emissions in international relations studies.

**Figure 5:** Trends in environmental nexus issues in major industrialized countries (2001–2019).

RETRACTED

**Figure 6:** Types of global environmental problems.

**Table 1:** Differences between the three international conventions on bills of lading.

	《Hague rule》	《Visby rules》	《Hamburg rules》
Liability of carrier	Imperfect liabilities for negligence (The so-called principle of negligence refers to the principle of responsibility if there is a fault and no responsibility if there is no fault. The civil law of general countries mostly adopts this principle as the basis).	No amendments were added	

The limitation of liability for carrier (from hague rules to hamburg rules, the maximum amount of compensation per unit of goods has been increased in turn)	The amount of compensation of the owner or carrier for loss of or damage to the goods or in connection with the goods shall not exceed £ 100 per piece or unit or the equivalent currency of £ 100.	Increase the maximum amount of compensation to 10000 gold francs per piece or unit or 30 gold francs per kilogram based on the gross weight of the lost or damaged goods, whichever is higher. At the same time, it is clear that a gold franc is a unit containing 66.5 mg of gold and 90 per 1000 purity	Increase the maximum liability of the carrier to 835 SDRs per package or freight unit or 2.5 SDRs per kilogram, whichever is higher.

Container	The goods are measured by each piece or unit, and the container problem is not specified	When the bill of lading indicates the number of packages or pieces of goods in the means of transport, each small piece of goods contained in the container or pallet shall be taken as the unit; when the bill of lading does not specify the specific number of goods, one container or one pallet shall be used as one piece of goods for compensation.	

**Table 2:** Classification of legal principles.

Classification criteria	Specific type
Content regulation	Authorized rules: A rule that stipulates that people have the right to do certain acts or not to do certain acts.
	Obligatory rules: Stipulate people's legal obligations, that is, the rules about what people should or should not do.
	Right meaning compound rule: Legal rules with the nature of granting rights and setting obligations.

The scope or degree of regulation and limitation of people's behavior	Mandatory rule: refers to the rule that the content provisions are mandatory and must be applied regardless of people's wishes.
	Arbitrary rules: Arbitrary rules are legal rules that allow people to choose or negotiate the contents of rights and obligations in legal relations within a certain range.

Degree of certainty of content	Certainty rule: it refers to the legal rule whose content has been clearly confirmed without invoking or referring to other rules to determine its content.
	Mandatory rules: Refer to the legal rules whose contents have not been determined, but only provide some general instructions, which shall be determined by the corresponding state organs through corresponding channels or procedures.

	Applicable rules: Refers to the rules that the content itself does not specify the specific behavior mode of people, and can be invoked or referred to other corresponding contents.

Functions of legal rules	Adjustment rule: a rule that adjusts an existing behavior.
	Constitutive rules: Rules that organize people to act according to the behavior stipulated in the rules.

RETRACTED

**Table 3:** International investment in funding for the global environment.

Item		2019
Number of environmental emergencies	(Times)	
Direct economic loss of environmental emergencies	(10000 yuan)	
Total investment in the treatment of environmental	(10000 yuan)	1036098.3
Investment in the urban environmental infrastructure	(10000 yuan)	515472.0
Gas supply	(10000 yuan)	26620.0
Centralized heating	(10000 yuan)	
Drainage works	(10000 yuan)	183607.0
Gardening and greening	(10000 yuan)	275858.0
Environmental sanitation	(10000 yuan)	29387.0
Investment in the treatment of industrial pollution	(10000 yuan)	96190.6
Waste water treatment	(10000 yuan)	52685.7
Waste gas treatment	(10000 yuan)	31900.0
Solid waste treatment	(10000 yuan)	6839.7
Noise treatment	(10000 yuan)	201.5
Other treatment	(10000 yuan)	4563.7
“Three simultaneities” environmental investment for	(10000 yuan)	424435.7

## Data Availability

The labeled dataset used to support the findings of this study are available from the author upon request.
